# A Novel Edge-Based Trust Management System for the Smart City Environment Using Eigenvector Analysis

**DOI:** 10.1155/2022/5625897

**Published:** 2022-05-26

**Authors:** G. Nagarajan, Serin V. Simpson, K. Venkatachalam, Adel Fahad Alrasheedi, S. S. Askar, Mohamed Abouhawwash, Parthasarathi P

**Affiliations:** ^1^Department of Computer Science and Engineering, Sathyabama Institute of Science and Technology, Chennai, India; ^2^Department of Computer Science and Engineering, SCMS School of Engineering and Technology, Kerala, India; ^3^Department of Computer Science and Engineering, CHRIST (Deemed to be University), Bangalore 560074, India; ^4^Department of Statistics and Operations Research, College of Science, King Saud University, Riyadh 11451, Saudi Arabia; ^5^Department of Mathematics, Faculty of Science, Mansoura University, Mansoura 35516, Egypt; ^6^Department of Computational Mathematics, Science, and Engineering (CMSE), Michigan State University, East Lansing, MI 48824, USA; ^7^Department of Computer Science and Engineering, Bannari Amman Institute of Technology, Erode, India

## Abstract

The proposed Edge-based Trust Management System (E-TMS) uses an Eigenvector-based approach for eliminating the security threats present in the Internet of Things (IoT) enabled smart city environment. In most existing trust management systems, the trust aggregation process completely depends on the direct trust ratings obtained from both legitimate and malicious neighboring IoT devices. E-TMS possesses an edge-assisted two-level trust computation approach for ensuring the malicious free trust evaluation of IoT devices. The E-TMS aims at removing the false contribution on aggregated trust data. It utilizes the properties of the Eigenvector for identifying compromised IoT devices. The Eigenvector Analysis also helps to avoid false detection. The analysis involves a comparison of all the contributed trust data about every single connected device. A spectral matrix will be generated corresponding to the contributions and the received trust will be scaled based on the obtained spectral values. The absolute sum of obtained values will contain only true contributions. The accurate identification of false data will remove the effect of malicious contributions from the final trust value of a connected IoT device. Since the final trust value calculated by the edge node contains only the trustworthy data, the prediction about the malicious nodes will be accurate. Eventually, the performance of E-TMS has been validated. Throughput and network resilience are higher than the existing system.

## 1. Introduction

A smart city environment has been established by utilizing the capabilities of edge computing-assisted IoT networks [1, 2]. The edge computing-assisted IoT network provides a collaborative computing facility with the help of a wide range of heterogeneous smart devices. Such a heterogeneous environment has the highest risk of being vulnerable to security attacks. Such networks require a robust trust management mechanism for maintaining a good device trust level. Trust management helps to keep users with increasing numbers. The traditional cloud-based trust evaluation approaches are incapable to analyze the context-aware trust relationships among connected IoT devices [3, 4]. The heterogeneity as well as the large size of the network became the prime reasons for the performance degradation of the centralized cloud servers. The centralized cloud server can work efficiently with smaller networks. But, it is hard to serve large-scale networks with centralized architecture. In such cases, the centralized server cannot offer real-time support to time-dependent applications. Also, it is not possible to make context-aware decisions for all the connected devices by a single cloud server.

Edge computing has been introduced to achieve context-aware data analysis among a large number of tiny IoT devices [5, 6]. The distributed architecture of edge computing-assisted networks is more vulnerable than the traditional cloud-based centralized architecture. Since the majority of the data will be processed near the end devices, the IoT network requires several data processing units (edge servers) at the edge of the network. That in turn increases the opportunities of the attackers to intrude on the network [7, 8]. All the security threats associated with the cloud server will be experienced at each tiny edge server. In other words, the attackers will utilize the vulnerabilities of edge servers to intrude on the network. Thus, the data aggregation process, as well as the control information management, must be done in a secure environment. The trust of each device and communication must be evaluated in regular intervals by using a robust trust evaluation framework. Thus, a scalability and mobility-aware universal trust mechanism needs to be incorporated with an IoT-enabled smart city environment. The paper mainly deals with the following aspects.

- Contributing a robust mechanism to evaluate the trustworthiness of smart city devices
- Contributing a two-level trust assessment approach for increasing accuracy
- A method for the direct assessment of device trust level based on the occurred events
- An event assessment approach for computing the trust value indirectly at the edge nodes
- Contributing an edge-driven Eigenvector-based approach for identifying the false trust contribution and malicious free aggregation of individual trust values
- Contributing an Eigenvector method to identify and isolate the malicious entities in the smart city environment

The following sections of this paper will give a detailed idea about the proposed E-TMS approach. The next section checks the requirement of a robust trust-based approach by analyzing the currently functioning approaches in IoT-enabled smart networks.  Section 3 gives an overview of the need for research in this area. The proposed Edge-based Trust Management System has been detailed in Section 4. The performance analysis and the comparative study have been included in Section 5. The conclusion and the future scope of research in this area have been discussed in Section 6.

## 2. Related Work

Wang et al. [9] introduced a recommendation-dependant system to take decisions for network management. The proposed work evaluates the trust of each entity in the smart city environment for excluding the malicious entities from the recommendation process. The computing node will accept the recommendations only from trustworthy IoT devices. The proposed work aims to utilize the trust-based recommendation mechanism to secure the network from various security threats. If the recommendation system considers only the trustworthy nodes, it can produce a reliable outcome. The proposed system evaluates each node based on the trust values. The trust will be calculated by the trust aggregation process. But the trust aggregation process does not possess an intelligent mechanism to eliminate the impact of malicious contributions. Thus, the selection of entities to participate in the recommendation system is vulnerable.

ElRahman and Alluhaidan [10] introduced a blockchain-based approach to secure healthcare IoT systems. The proposed framework designs a trust model to prevent data leakage. Most of the data involved with the healthcare systems will be related to personal health information. Such sensitive data needs to be handled carefully. The proposed system initially builds ontologies for the IoT network. The ontology-based IoT-enabled healthcare system utilizes semantic references to find cognitive relationships. Upon creating the ontologies, the framework applies blockchain technologies to secure the IoT network. Blockchain technology offers sensor data integrity to the perception layer, authentication service to the network layer, privacy-preserving schemes to the middleware layer, and mechanisms to ensure the overall security of the devices in the application layer. The overall operational complexity of the proposed approach is quite high. To enhance the performance of the edge servers, it is always adequate to employ only lightweight algorithms.

Adewuyi et al. [11] designed a recommendation dependant approach to evaluate the network entities. The system receives recommendations from all the registered entities to finalize the recommendation trust. Upon finalizing the recommendation trust, the proposed framework applies the belief function to estimate the trustworthiness of the evaluated trust. The output of the belief function indicates the willingness of each node to trust the recommendation trust. Thus, the nodes need not blindly believe the recommendations. Each node will act based on the output of the belief function. Thus, the recommendation trust cannot make changes directly to the existing trust relationships. Since the recommendation trust also includes the contribution from malicious nodes, the evaluation performed by the belief function may not be accurate always.

Fang et al. [12] introduced a fog-based approach for ensuring data integrity. The proposed method uses a source anonymity algorithm to make the source node undetectable to malicious nodes. Also, it integrates RSA digital signature to preserve the confidentiality of data. It follows a randomly delayed transmitting scheme to reduce energy consumption. But the overall framework lacks an intelligent approach to isolate the involvement of malicious nodes from the execution of subsidiary methods. Manimurugan et al. [13] introduced a machine learning-based approach for detecting malicious nodes. The work has been introduced to prevent unauthorized access to network resources. The method evaluates each entity by gathering necessary information from the neighboring nodes. The Deep Belief Network predicts the behavior of each network entity by analyzing the individual contributions. Since the mechanism accepts trust contributions also from malicious nodes, the malicious node can make a large impact on the output. By utilizing this limitation, a malicious node can continue in the network for a long period.

Most of the trust management mechanisms in the IoT platform mostly adopt the contributive approach which accepts the recommendations from both legitimate and malicious nodes. All those systems are not concerned about malicious contributions. Such malicious contributions can mislead the network.

## 3. Problem Statement and System Architecture

A smart city environment holds several heterogeneous tiny end devices. Due to economic constraints, it is not possible to deploy resource-rich devices at the bottom layer to execute complex computations [14, 15]. Thus, a smart city environment highly relies on cloud/edge paradigms to fulfill both its operational and security needs [16, 17]. In most of the existing trust evaluation mechanisms, the edge server will aggregate the trust information from the connected IoT devices. But, the existing mechanisms usually do not possess an intelligent method to identify and eliminate the false contribution from the malicious nodes. This work mainly aims at identifying such untrustworthy contributions. The overall trust in E-TMS will be computed by considering the individual trust values obtained from direct as well as indirect evaluations. The direct trust will be obtained from the neighboring nodes based on the node's behavior toward a set of network events. The indirect trust will be computed depending on the node's involvement in network management. E-TMS performs an Eigenvector Analysis on the aggregated final trust values to detect the misleading contributions. The proposed two-level evaluation approach could produce the exact reflection of a node's behavior on the final trust value. Based on those observations, an edge node can confirm the malicious behavior of a connected device.

The architecture of the proposed E-TMS is shown in Figure 1. The cloud data center is responsible for performing all the complex computations. The edge nodes will be placed near the end devices. The edge node can fulfill all the required real-time computational needs of the smart city environment. The end devices will perform the individual trust assessments about the neighboring nodes and the edge servers will aggregate the same. The edge servers are also responsible for identifying and eliminating malicious contributions. The proposed architecture balances the computational overload of both cloud servers and the end devices by placing the real burden on the edge servers. A detailed report will be shared with the cloud server, whenever it is required.

## 4. Proposed System

E-TMS uses Eigenvector-based malicious identification approach for identifying and eliminating the malicious nodes from the smart city environment. The trust management system proposed in E-TMS uses a two-level trust assessment approach for generating the final trust about a node.

- Level 1: Edge Independent Direct Assessment
- Level 2: Edge-Based Indirect Assessment

The final event-based trust values will be sent to the edge node for performing the Eigenvector computations to remove false contributions. The nodes which contribute malicious data will be included in the Do-not-Consider-List (DCL) and all the listed malicious entities will not be further considered.

**Definition 1 .**

(trustworthy node). The trustworthy node will behave legitimately to all the network events. Such a node will do its best to avoid packet drops and forward each packet to the desired next hop. A trustworthy node will hold the latest DCL packet, and all the routing decisions will be carried out only based on the available information in the DCL. Such nodes will strictly follow the rules associated with the node joining procedure. Also, the trustworthy node will perform all the optimizations required for maintaining the residual energy at a satisfying level. Any malicious interruptions can mislead the network entities from the above etiquettes. A trustworthy node must be able to withstand all such malicious interventions.

### 4.1. Event-Based Trust Assessment

All nodes in the network will compute event-based trust (ET_ij_) about all other nodes in their occupying cluster. All such assessed values along with their own self-assessed score will be sent to the edge node for identifying the malicious nodes. The event-based trust assessment involves two levels, edge independent direct assessment and edge-based indirect assessment. Both assessments will consider different network events for computing the trust score.

#### 4.1.1. Edge Independent Direct Assessment (Level 1)

All nodes will compute the event-based direct trust (*DT*_*ij*_) of their neighboring nodes and that will be saved in the Local Trust Table (LTT).

**Definition 2 .**

(direct trust). It can be defined as the trustworthiness of that node toward the neighboring nodes. A neighboring node can compute the same by considering all the events occurring directly between them. The predicted response for every event will be identified at the initial level. The neighboring node will observe the evaluating node for a certain period. All the responses of the observed node for the occurring events will be examined closely. The prioritized or nonprioritized score can be assigned to all the responses. Direct trust can be formulated based on the obtained score values.

The direct trust can be computed using

(1) $$\begin{array}{c} DT_{ij}=\frac{{\text{DirectTrustScore}}_{\text{ij}}}{\text{TotalnumberofEventsConsidered}}. \end{array}$$

The events considered for calculating the direct trust have been selected based on data transmission, DCL distribution, neighbor discovery process, and path determination. The events associated with the above-mentioned actions have been listed in Table 1. All the events which can produce a significant impact on results are considered for the direct trust evaluation. The events which have occurred in the desired fashion will contribute a positive score to the direct trust evaluation, and all undesired events will contribute a negative score. The initial Direct Trust Score will be assigned as “0” for newly joined nodes. Based on the involvement in the network, the Direct Trust Score of a neighboring node will be incremented or decremented by the assessing node.

The following events will be considered by node “*n*_*i*_” during the direct assessment of neighboring node “*n*_*j*_”.

The Local Trust Table will be shared with the edge node, and further updates will be communicated at regular intervals. Based on the same, the edge server will construct a Global Trust Table (GTT) where each column represents the direct trust about a single node contributed by the neighboring nodes.

#### 4.1.2. Edge-Based Indirect Assessment (Level 2)

The node “*n*_*i*_” will compute the event-based indirect trust of other cluster members by considering some network events. The events considered for the calculation of indirect trust have been listed in Table 2.

Node movement, node joining procedure, residual energy, and acknowledgment process have been considered for calculating the indirect trust. The neighboring node will compare the residual energy with a value that has been explicitly derived based on the application, to determine the score (+1 or a −1). Since the data about all the above-listed events are obtained from the edge node, the assessment is considered an indirect assessment.

**Definition 3 .**

(indirect trust). The indirect trust of a node can be defined as the measure of desirability in general network events. A node can calculate the indirect trust of its neighboring nodes by obtaining the necessary information from the monitoring authority (connected edge node). All the general network events can be considered for this evaluation. Since a normal network entity does not have access to the log data of general events, the data need to be obtained from the connected edge node. Thus, the evaluation completely depends upon the data provided by a third entity. Thus, the evaluation has been termed an indirect evaluation.

The event-based indirect trust (*IT*_*ij*_) of node “*n*_*j*_” can be computed using

(2) $$\begin{array}{c} IT_{ij}=\frac{{\text{IndirectTrustScore}}_{\text{ij}}}{\text{TotalnumberofEventsConsidered}}. \end{array}$$

Both direct trust and indirect trust are equally significant while computing event-based trust.

#### 4.1.3. Event-Based Trust (*ET*_*ij*_)

In order to calculate the event-based trust, the direct trust values (*DT*_*ij*_) about the assessed node (*n*_*j*_) will be obtained from the GTT. The edge node will send the values listed in the column corresponding to the assessed node. After getting the direct trust values, the assessing node (*n*_*i*_) will do the following computations to nullify the effect of malicious contributions.

(3) $$\begin{array}{c} \text{Avg}=\sum_{i=1}^{m}DT_{ij}. \end{array}$$

As an initial step, the average value of all the received direct trust values about node “*n*_*j*_” will be computed. It includes the contributions from “*m*” contributing nodes that have the direct connectivity (neighbors) with node “*n*_*j*_”. The deviation of each Direct Trust Value from the average value will be computed and listed as follows:

(4) $$\begin{array}{c} {\text{dev}}_{ij}=\left|\text{Avg}-DT_{ij}\right|. \end{array}$$

(5) $$\begin{array}{c} \text{DeviationList}=\;\left({\text{dev}}_{1\text{j}}{\text{,dev}}_{2\text{j}}{\text{……dev}}_{\text{mj}}\right) \end{array}$$

The largest deviation value among the obtained deviations can be represented as *LD*. The weight values for nullifying the effect of malicious contributions can be computed using the following equations:

(6) $$\begin{array}{c} {\text{diff}}_{ij}=\left|\left(L\;D+0.001\right)-{\text{dev}}_{ij}\right|. \end{array}$$

(7) $$\begin{array}{c} \text{DifferenceList}=\;\left({\text{diff}}_{1j},\text{diff}\ldots \ldots {\text{diff}}_{mj}\right). \end{array}$$

(8) $$\begin{array}{c} \text{Avg.Difference}=\;\frac{\sum_{i=1}^{m}{\text{diff}}_{ij}}{m}. \end{array}$$

(9) $$\begin{array}{c} \text{WeightValue},\;w_{ij}=\frac{{\text{diff}}_{ij}}{\text{Avg.Difference}}. \end{array}$$

The received direct trust values will be multiplied with the corresponding weight values, and the average of obtained results will be the malicious free average of received direct trust values (MFDT_*ij*_) about node “*n*_*j*_”:

(10) $$\begin{array}{c} {\text{MFDT}}_{ij}=\frac{\sum_{i=1}^{m}DT_{ij}\times w_{ij}}{m}. \end{array}$$

Thus, the malicious contributions cannot tamper with the individual trust assessment process. The node “*n*_*i*_” can compute the final event-based trust (ET_*ij*_) of node “*n*_*j*_” using equation (12):

(11) $$\begin{array}{c} ET_{ij}=0.5\times IT_{ij}+0.5\times {\text{MFDT}}_{ij}. \end{array}$$

Each node will assess the event-based trust value of all the nodes in the same cluster. The obtained results will be shared with the connected edge server. Further, a trust aggregation process will be carried out at the edge server to examine the malicious behavior. Since the malicious nodes are also allowed to send the trust values, the edge server needs to be more efficient to identify the malicious contributions.

### 4.2. Trust Aggregation

Both trust aggregation and the process of finding the malicious nodes will be done at edge nodes for reducing the computational overhead at individual IoT devices. The received event-based trust will be stored as a (*n* × *n*) matrix (RT) at the edge node:

(12) $$\begin{array}{c} RT=\left[\begin{array}{cccc} ET_{\left(1,1\right)} & ET_{\left(1,2\right)} & \ldots & ET_{\left(1,n\right)}\\ ET_{\left(2,1\right)} & ET_{\left(2,2\right)} & \ldots & ET_{\left(2,n\right)}\\ \cdot & \cdot & \cdot & \cdot \\ \cdot & \cdot & \cdot & \cdot \\ ET_{\left(n,1\right)} & ET_{\left(n,2\right)} & \ldots & ET_{\left(n,n\right)} \end{array}\right]. \end{array}$$

The *i*^th^ row of matrix RT includes the trust contributions of “*n*” number of cluster members about *i*^th^ IoT device. Similarly, the column of matrix RT includes the trust contributions of a single IoT device in the cluster about all other cluster members. Thus, the row average of matrix RT represents the relative trust of a single IoT device.

(13) $$\begin{array}{c} {\text{RelativeTrust}}_{i}=\;\frac{\sum_{j=1}^{n}ET_{\left(i,j\right)}}{n}. \end{array}$$

The relative trust includes the contribution from both legitimate as well as malicious nodes. Thus the edge node cannot conclude the malicious behavior of a cluster member simply based on the row average value/relative trust. Thus, an Eigenvector-based malicious node identification approach has been introduced in the next section.

### 4.3. Eigenvector-Based Malicious Node Identification

The effect of trust contributions from the malicious nodes needs to be nullified for getting the actual trust value of individual cluster members. Here, we are applying a vector-based malicious identification approach for excluding the false trust contribution from the malicious nodes. We consider each trust contribution as an independent vector. In order to construct orthogonal vectors, the input matrix must be a symmetric matrix. Thus, it is required to construct a real symmetric matrix corresponding to the matrix RT. The device trust values received about a single node and the device trust values contributed by a single node will possess some unique patterns. Thus, the symmetric matrix must be capable enough to hold all such properties of the parent matrix (RT). The covariance matrix of any matrix will be symmetric. The covariance matrix is defined as a matrix that is able to show the covariance between each pair of elements in a matrix. The covariance matrix of RT can be represented as follows.

(14) $$\begin{array}{c} CoRT=\left[\begin{array}{cccc} {\text{CoRT}}_{\left(1\text{,}1\right)} & {\text{CoRT}}_{\left(1\text{,}2\right)} & \ldots & {\text{CoRT}}_{\left(1\text{,n}\right)}\\ {\text{CoRT}}_{\left(2\text{,}1\right)} & {\text{CoRT}}_{\left(2\text{,}2\right)} & \ldots & {\text{CoRT}}_{\left(2\text{,n}\right)}\\ \cdot & \cdot & \cdot & \cdot \\ \cdot & \cdot & \cdot & \cdot \\ {\text{CoRT}}_{\left(\text{n,}1\right)} & {\text{CoRT}}_{\left(\text{n,}2\right)} & \ldots & {\text{CoRT}}_{\left(\text{n,n}\right)} \end{array}\right]. \end{array}$$

where CoRT_(*i,j*)_ will be same as CoRT_(*j,i*)_ for all *i* ≠ *j*. As per the probability theory and statistics, the diagonal elements of the covariance matrix (CoRT) can be computed using equation (16).

(15) $$\begin{array}{c} {\text{CoRT}}_{\left(i,j\right)}=\left(\frac{1}{n}\overset{n}{\underset{i=1}{\sum }}ET_{\left(i,j\right)}^{2}\right)-{\left(\frac{1}{n}\overset{n}{\underset{i=1}{\sum }}ET_{\left(i,j\right)}\right)}^{2}. \end{array}$$

Also, the covariance of nondiagonal elements will be computed using equation (17).

(16) $$\begin{array}{c} {\text{CoRT}}_{\left(i,j\right)}=\frac{1}{n}\left(\sum_{k=1}^{n}ET_{\left(k,i\right)}ET_{\left(k,j\right)}\right)-\left(\sum_{k=1}^{n}ET_{\left(k,j\right)}\right). \end{array}$$

Since each element in the covariance matrix has been computed by considering the covariance of each element in the matrix with other elements, all the properties of the parent matrix will be cloned effectively to the resulting matrix (CoRT). The Eigenvector and spectral values corresponding to the trust values received from the cluster members can be computed as follows. The characteristic equation can be represented as

(17) $$\begin{array}{c} \left|\text{CoRT}-\lambda I\right|=0, \end{array}$$

where “CoRT” is an (*n* × *n*) matrix. “*λ*” represents the spectral values corresponding to the trust values received from a single node. “I” represents the identity matrix in the order of “CoRT”. The characteristic equation (17)will be *n*^th^ degree polynomial in “*λ*”. While solving (17), we will get “*n*” spectral values {*λ*_1_, *λ*_2_,…, *λ*_*n*_}. The linear homogeneous system with respect to the (17) can be represented as

(18) $$\begin{array}{c} \left(CoRT*X-\lambda *X\right)=0\\ CoRT*X=\;\lambda *X, \end{array}$$

where *X* is an (*n* × 1) column matrix and *X* ≠ 0 (i.e, nonzero vector). The matrix “*X*” is known as Eigenvector. Since the multiplication with identity matrix results in the same value, *λ* in equation (19) can be represented as a product of “*λ*” and “*I*”.

(19) $$\begin{array}{c} \left(CoRT-\lambda *I\right)\;X=0,\\ \left(CoRT*X-\lambda *\text{I}*\text{X}\right)=0. \end{array}$$

We can solve the above-mentioned linear system (19) corresponding to each value of “*λ*”. While solving the same for each value of “*λ*”, we will get a nonzero Eigenvector (*X*_*i*_) with order (*n* × 1). A spectral matrix can be constructed by including each “*X*_*i*_”, corresponding to all *λ* values.

(20) $$\begin{array}{c} \text{Spectral Matrix},\text{SM }=\left[{\text{X}}_{1},{\text{X}}_{2}\ldots \ldots \ldots {\text{X}}_{\text{n}}\right]. \end{array}$$

Here, *X*_*i*_ represents the Eigenvector corresponding to “*λ*_*i*_”.

(21) $$\begin{array}{c} X_{i}=\;\left[\begin{array}{c} v_{\left(1,i\right)}\\ v_{\left(2,i\right)}\\ \cdot \\ \cdot \\ v_{\left(n,i\right)} \end{array}\right]. \end{array}$$

The spectral matrix can be expanded by substituting the values for *X*_1_ to *X*_*n*_. The spectral matrix of order (*n* × *n*) after substituting the individual values is shown in

(22) $$\begin{array}{c} SM=\left[\begin{array}{cccc} v_{\left(1,1\right)} & v_{\left(1,2\right)} & \ldots & v_{\left(1,n\right)}\\ v_{\left(2,1\right)} & v_{\left(2,2\right)} & \ldots & v_{\left(2,n\right)}\\ \cdot & \cdot & \cdot & \cdot \\ \cdot & \cdot & \cdot & \cdot \\ v_{\left(n,1\right)} & v_{\left(n,2\right)} & \ldots & v_{\left(n,n\right)} \end{array}\right]\;, \end{array}$$

where *v*_(1,1)_ represents the *i*^th^ Eigenvector value corresponding to the *i*^th^ spectral values (*λ*_*j*_). A transformation process has been applied to the CoRT matrix for getting the SM matrix. It is a process of scaling the received trust value corresponding to the obtained spectral values. The obtained values inside the spectral matrix represent the direction of each individual trust data. The mathematical operations applied to the received trust eliminate the effect of malicious contribution. Absolute row sums of the spectral matrix are the malicious free scalar values (MFSVs) of received trust corresponding to individual nodes.

(23) $$\begin{array}{c} {\text{MFSV}}_{i}=\sum_{j=1}^{n}\left|v_{\left(i,j\right)}\right|, \end{array}$$

where MFSV_i_ represents the malicious free scalar values of *i*^th^ node. The row average (RA_*i*_) of obtained MFSV_*i*_ value represents the actual trust value of *i*^th^ node.

(24) $$\begin{array}{c} {\text{RA}}_{i}=\;\frac{{\text{MFSV}}_{i}}{n}. \end{array}$$

The RA_i_ represents the aggregated trust of *i*^th^ node, which has been evaluated by considering the contributions of “*n*” number of nodes. The Eigenvector-based operations on received trust remove the effect of malicious trust contributions from the compromised nodes. Since the aggregated trust value of *i*^th^ node (RA_*i*_) contains only the true trust contributions, the RA_*i*_ value can be used for the detection of malicious nodes inside the network. An Aggregated Trust Threshold (ATT) has been fixed to 0.2 based on the repeated simulation results for identifying the malicious nodes inside the network. Nodes having RA_*i*_ value less than ATT can be marked as malicious and will be included in DCL. The updated DCL packet will be circulated among the network entities at a regular time interval. Thus, the local copies of DCL stored at each network entity will be replaced with the updated list without any delay. A legitimate network node will initiate a communication only after verifying the trustworthiness of the recipient entity with the DCL stored in the local memory. This approach will eliminate the chances of the inclusion of malicious nodes in new communication. Thus, the proposed method can ensure the complete isolation of malicious nodes with the help of DCL.

## 5. Comparison and Analysis of Experimental Results

The performance of E-TMS has been examined with the help of network simulator NS 2.35.  Table 3 summarizes the network conditions introduced for setting up the simulation environment. Since the IoT devices are mobile in the network field, the direction of the signals cannot be predicted. Thus, the antenna must have the ability to accept the signals in 3600. Thus, the simulation environment uses an omnidirectional antenna in the physical layer. In real-time systems, the use of an omnidirectional antenna increases the possibility of receiving interferences from all directions. Due to this reason, performance degradation may be experienced in real-time systems.

The experimental setup examines the performance of the proposed method in two different aspects. Initially, the performance metrics have been calculated with respect to varying network load (as mentioned in scenario 2 under Table 3). Further, the evaluation proceeds with a constant network load for a different number of nodes in the same network field (as mentioned in scenario 1 under Table 3). The second evaluation environment has been introduced to study the behavioral changes of E-TMS under different network conditions. In order to compare the obtained results, the works, SAODV [18], SLICER-TMU [19], SAL-SAODV [12], and DBNIDS [13] have also been evaluated under the same network conditions. The efficiency has been evaluated based on average throughput, network resilience, and packet delivery ratio (PDR) [20–22]. The throughput can be defined as the number of successful receptions during a stipulated interval. The resilience value is a ratio of unsuccessful packet deliveries and the number of initiations. It gives the exact measure of unsuccessful packet delivery attempts. PDR is the measure of successful packet deliveries with respect to the total communication initiations in a stipulated time interval.

The average throughput under the varying number of nodes and varying network load has been evaluated and plotted in Figures 2 and 3 It is the count of successfully received packets at the receiver side. E-TMS could achieve better throughput by the proper identification of malicious nodes in both scenarios.

Figures 4 and 5 represent the network resilience assessed in both scenarios. E-TMS utilizes the features of Eigenvector for identifying the malicious trust data contributions during the trust aggregation process. The proper isolation of compromised entities will avoid the chances of having unsuccessful communication links. The lower resilience of E-TMS indicates that only a minimal number of compromised communications has been experienced during the assessed time interval.

The packet delivery ratio (PDR) based comparison under scenario 1 has been plotted in Figure 6. A better packet delivery ratio can be achieved only when the network becomes malicious-free. A good trust management system can ensure the trustworthiness of the network. The proposed E-TMS experiences a linear decrease in PDR under the given network conditions. But, it could maintain higher PDR by the incorporation of a two-level event-based trust assessment mechanism.

Figure 7 shows the PDR of 5 works based on the varying network load. The network load has been increased to 6000 kb. E-TMS maintains a stable packet delivery ratio even with the higher load. By incorporating a good load balancing mechanism, the network can withstand the burden of a higher load. But, the attacks from maliciously compromised nodes will destroy the harmony between the increased load and packet delivery. E-TMS could ensure a good PRD count by removing all the impurities from the network. Further findings of E-TMS over the existing works have been included in Table 4.

The existing approaches for trust data aggregation fail to identify the malicious contributions. Such contributions have the capacity to mislead the network [23–29] if the network does not possess an intelligent approach to identify the same. The proposed E-TMS approach has the ability to remove malicious contributions. Thus, it could outperform the existing approaches in identifying the maliciously compromised nodes. The experimental result justifies the above statement.

## 6. Conclusion

The proposed trust management system, E-TMS, addresses the issues associated with Direct Trust Management Systems. Both legitimate and malicious nodes will contribute the trust data about their neighboring nodes. The aggregated trust value about a node may become inaccurate due to the presence of malicious contributions. E-TMS uses an Eigenvector-based approach for eliminating the malicious contributions while aggregating the individual trust contributions about a node. Rather than completely depending on the direct assessment, E-TMS possesses a two-level trust evaluation approach by considering both direct trust and indirect trust. As per the experimental results, E-TMS could outperform other existing trust management systems by the proper identification and elimination of malicious contributions, emerging from maliciously compromised nodes. In the future, a real-time trust management system can be developed using a machine learning system.

## Figures and Tables

**Figure 1:** System architecture.

**Figure 2:** Average throughput (scenario 1).

**Figure 3:** Average throughput (scenario 2).

**Figure 4:** Network resilience (scenario 1).

**Figure 5:** Network resilience (scenario 2).

**Figure 6:** Packet delivery ratio (scenario 1).

**Figure 7:** Packet delivery ratio (scenario 2).

**Table 1:** Event-based score allotment: direct trust.

Events	Score
Correct forwarding of the offered packet	+1
Dropping an offered packet	−1
Reception of updated DCL packet from “*n*_*j*_”	+1
Reception of old DCL broadcast form “*n*_*j*_”	−1
Timely reply for a hello packet	+1
Route request for a node listed in DCL	−1

**Table 2:** Event-based score allotment: indirect trust.

Events	Score
Leaving a cluster without notifying the edge node	−1
Leaving the cluster in a proper way	+1
Violation of node joining procedure	−1
Approved node joining	+1
Residual energy	−1 or +1
Based on acknowledgment	−1 or +1

**Table 3:** Simulation parameters.

Parameters		Scenario 1	Scenario 2
Physical layer	S. propagation	Two-ray ground	
	Antenna model	Omniantenna	

Mac layer	Mac protocol	802.11	
	Link bandwidth	1 MB	

Simulation	Size of network field	1000 m × 1000 m	1000 m × 1000 m
	Rate (Mbs)	0.1	0.1
	Packet size (B)	1000	1000
	Traffic type	CBR	CBR
	Duration (s)	600	600
	Speed (m/s)	25	25
	Number of nodes	25/50/75/100/125	100
	Load	500 Kb	1000–6000 Kb

Queue	Type	DropTail/PriQueue	
	Size	50	

NS2 version		2.35	
Processor		Intel processor 3 GH	
Operating system		Ubuntu 16.04 LTS	

**Table 4:** Analysis of proposed work.

Work name	Significance	Methodology for identifying the malicious trustdata contributions	Methodology	Significance/limitations
E-TMS	(i) Eigenvector-based approach for eliminating the malicious contributions	Present	(i) Malicious free aggregated trust value evaluation	(i) Two-level trustevaluation approach
SAODV [18]	(i) Resistant toward routing attacks	Nil	(i) Enhancement of path determination	(i) Introduced only to secure AODV
SLICER-TMU [19]	(i) Prevention of identity-based attacks	Nil	(i) Secure authentication mechanism	(i) Vulnerable to malicious trust contributions
SAL-SAODV [12]	(i) Power-aware approach	Nil	(i) Architectural enhancement	(i) Fog-based approach
DBNIDS [13]	(i) Malicious attack detection	Nil	(i) Deep belief neural network-based approach	(i) Method accepts trust data contributions from both malicious as well as legitimate nodes

## Data Availability

All the required data used to support the findings of the study are available within the article.
